The article "Perspectives of Molecular Therapy-Targeted Mitochondrial Fission in Hepatocellular Carcinoma" was retracted in 2024. Reasons: signs of a paper mill; compromised peer review; unreliable results or conclusions.

# Perspectives of Molecular Therapy-Targeted Mitochondrial Fission in Hepatocellular Carcinoma

**DOI:** 10.1155/2020/1039312

**Published:** 2020-12-29

**Authors:** Hanwen Zhang, Yanshuo Ye, Wei Li

**Affiliations:** Department of Hepatobiliary-Pancreatic Surgery, China-Japan Union Hospital of Jilin University, Changchun 130033, China

## Abstract

Current advances of molecular-targeting therapies for hepatocellular carcinoma (HCC) have improved the overall survival significantly, whereas the results still remain unsatisfied. Recently, much attention has been focused on organelles, such as the mitochondria, to reveal novel strategies to control the cancers. The mitochondria are vital organelles which supply energy and maintain metabolism in most of the eukaryotic cells. They not only execute critical bioenergetic and biosynthetic functions but also regulate ROS homeostasis and apoptosis. Existing in a dynamic equilibrium state, mitochondria constantly undergo the fission and fusion processes in normal situation. Increasing evidences have showed that mitochondrial fission is highly related to the diseases and cancers. Distinctive works have proved the significant effects of mitochondrial fission on HCC behaviors and the crosstalks with other molecular pathways. Here, we provide an overview of the mitochondrial fission and the link with HCC, emphasizing on the underlying molecular pathways and several novel materials that modulate HCC behaviors.

## 1. Introduction

Hepatocellular carcinoma (HCC) constitutes 80-90% of primary liver cancers. It is the second most frequent cause of cancer-related death all over the world [1, 2]. Although various techniques have long been applied to treat HCC, poor earlier diagnosis rate and high risk for recurrence are still significant problems puzzling scholars [3]. Nowadays, with the development of biological and medical sciences, the new medical treatment strategies depend on the molecular pathways significantly. Molecular-targeted agents are extensively used in systemic therapy currently for HCC by targeting multikinases or receptors for vascular endothelial growth factor. Sorafenib has been used as the first-line multitarget drug for HCC whereas inefficient therapy attributed to drug resistance still remains to be an unresolved problem [4, 5].

On the basis of the development of morphometric methods and seminal researches of untrastructure of HCC in the 1980s [6, 7], morphological and functional change of organelles such as the mitochondria is drawing people's attention. The potential roles of mitochondria in the proliferation and survival of tumor cells are raising more concerns recently. Mitochondria are considered pluripotent organelles, generating ATP, producing and eliminating ROS, and controlling apoptosis of the cells [8]. Besides, the mitochondria engage in highly dynamic state, including fission and fusion. It is a very important process for the mitochondria which undergo such a balanced process in maintaining a healthy mitochondrial population and functions, and the ubiquitous and fundamental processes serve as important biomarkers for detection of diseases [9]. Moreover, mitochondrial dynamics play important roles in oxidative phosphorylation (OXPHOS) through regulating mtDNA, facilitates mitochondrial morphology, transport, mitophagy, and apoptosis [10]. Therefore, any functional or morphological alteration of mitochondria may affect hepatocarcinogenesis as they are major organellar regulators of cell metabolism.

Despite the vital contributions to cell life and metabolism, mitochondria underpin several diseases such as neurodegenerative disorders, cardiovascular diseases, and cancers [11]. It has been reported that the function disorder is related to cancers in the past, but dynamics changes and the underlying molecular pathways alterations are coming into sight as novel diagnostic targets in recent years. Dysregulation of dynamin-related protein 1 (Drp1), which mediated the mitochondrial fission, might lead to the resistance to apoptosis, increased proliferation, and invasiveness of cancers. Accumulating evidences verify a link between enhanced expression of Drp1 and HCC in the dynamic change of the mitochondria [12], suggesting a novel pathway to cure HCC and prevent the recurrence and metastasis. Here, we provide an overview on the recent update by presenting new insights into targeting molecular pathways such as Drp1, Ca2+ pathway, and MTP18 to inhibit mitochondrial fission-related hepatocarcinogenesis with an emphasis on the underlying mechanisms.

## 2. Mitochondrial Fission

### 2.1. Machinery of Mitochondrial Fission

The Drp1 is a GTPase that serves as the master regulator in mitochondrial fission. Similar to other dynamin family members, such as homolog Dnm1 in yeast, it contains an N-terminal GTPase, a middle domain, an additional alternatively spliced brain-specific isoform (human-specific), and a C-terminal GTPase effector domain involved in self-assembly [13–15]. Much of Drp1 resides in cytosol unless is recruited by proteins which is assembled on the mitochondrial outer membrane (MOM), including Fis1, MFF, MiD49, and MiD51 [9]. Fis1 and MFF play key roles in the interaction with Drp1, mainly performing the recruitment function [16, 17]. MiD49/51 use to be referred as SMCR7 and SMCR7L proteins and are renamed mitochondrial dynamic proteins of 49 kDa (MiD49) and 51 kDa (Mid51) because of their mitochondrial activity and size [18]. Those are considered to be new components in the directing of the Drp1 to mitochondrial surface, but the mechanisms still remain to be further studied [18, 19]. Knockdown or reduction of any of these proteins will result in the disorder of mitochondrial dynamic.

### 2.2. Mechanism of Mitochondrial Fission

Mitochondrial fission is a complicated process begins with the recruitment of Drp1 to the mitochondria executed by MOM proteins Fis1, MFF, MiD49, and MiD51 [19, 20]. The endoplasmic reticulum (ER) is one of the organelles that can contribute to Drp1 recruitment through contacting with mitochondria, which are referred to as mitochondria-associated membrane (MAM). MAM facilitates the transformation of Ca^2+^, a core component of calcium pathway that promotes mitochondrial fission [21]. Once Drp1 binds to receptors located in MOM, a functional oligomer forms and transports to where the fission occurs [22]. The oligomerization process is similar to classical dynamins in vesicular budding pathways that Drp1 assembles into higher-order structures, forming rings and spirals around the mitochondria, further constricting the mitochondrial tubule and severing the mitochondrial membranes through GTP hydrolysis [9, 15] (Figure 1).

## 3. Mitochondrial Dynamics and Cancers

### 3.1. Functions of Mitochondrial Fission

The mitochondria undergo dynamical changes between fusion and fission to stabilize the morphology and avoid fragmentation and elongation due to unbalanced fission and fusion [23]. Notwithstanding controlling the shape, mitochondrial fission also plays important roles in diverse cellular events. For instance, mitochondrial fission is linked to embryonic development. Reduced neurites and defective synapse formation were observed by knocking out Drp1 in mice, suggesting the essential role in mitochondrial fission in the development of the nervous system [24]. Fission is also demonstrated to be linked to the mitochondrial inheritance and facilitating segregation as well as the mitochondrial homogenization during cell division [25]. Thus, the regulatory effect of mitochondrial fission on the release of intermembrane-space proteins into the cytosol contributes to apoptosis [26]. However, in spite of much outstanding works having been revealing biological functions of mitochondrial fission, the molecular/organellar networks and intricate functions of mitochondrial fission have not yet been fully characterized.

### 3.2. Dysfunctions of Mitochondrial Fission and Cancers

As a major metabolism regulating organelle in cells, dysfunctions of the mitochondria can result in a variety of diseases. Although dysfunctions of signaling pathway such as PI3K/AKT and MAPK, and their crosstalks, have been widely considered to take major responsibility for the development of several kinds of cancers for decades [27, 28], dysfunctions of mitochondrial fission are recently brought to the forefront along with in-depth researches. Most of the mitochondrial proteins are encoded with nuclear DNA, but a small fraction of which are encoded by mitochondrial DNA (mtDNA) [29]. Mutation in mtDNA may result in a wide range of cell dysfunctions or metabolism alterations such as excessive reactive oxygen and abnormal calcium homeostasis [29]. These have laid the foundation of the considerable possibility to explain the potential roles of abnormal mitochondrial behaviors in the process of carcinogenesis and to facilitate clinical examination and cancer diagnosis.

Many studies have reported that the increases of mitochondrial fission is possibly protumorigenic and is associated with oncogene expression, metabolism, cell behaviors, and stress responses [30, 31]. Cancer cells can be characterized by distinguishing features, one of which is their ability to proliferate infinitely along with dysregulation of cell cycles that equips cancer cells with replicative “immortality” [32]. Moreover, cancer cells also escape from microphage-mediated destruction including phargocytosis in the tumor microenvironment (TME), along with mitochondrial fission during neoplastic transformation [33]. The other distinct feature of cancer cells is uncontrolled proliferation during neoplasia, along with deviant Drp1 phosphorylation at Ser616 driven by CDK1/cyclin B [33]. Mitochondrial fission also plays an important role in cell division. The mitochondria undergo dynamic changes of membranes and are transmitted to daughter cells in a Drp1-dependent manner. In Drp1 knockdown HeLa cells, the maintainaA(mtDNA) into cytosol, which promotes the CCL2 mediated-recruitment of tumor-assnce of tubular mitochondrial structures, is observed, thus leading to the reduction of mitochondrial fragmentation during mitosis [34]. Moreover, mitochondrial fission is found to facilitate promoted migration of cancer cells. Silencing endogenous Drp1 by transfecting Drp1-targeting siRNAs can downregulate migration and invasion of breast cancer cells. Drp1 inhibitor Midiv1 treatment can produce the same effect [35]. A recent study reports that the increased mitochondrial fission lead to the release of mitochondrial DNociated microphage (TAMs) and enhances HCC progression [36, 37]. In brief, mitochondrial fission participates in tumor progression at various aspects. Of note, studying of mitochondrial dynamic works in cancer cells via ultrastructure level has become quite complex, and what is happening in this ubiquitous process is still a matter of controversy. Elaborate description of molecular networks that modulate different cancer cell behaviors will provide a significant guidance in further studies.

## 4. Molecular-Targeted Therapies on Mitochondrial Fission-Related Pathways

### 4.1. Mdivi-1

Mdivi-1 is a cell permeable quinazolinone that inhibits mitochondria fission in both yeast and mammalian cells. There are more than 126 primary research publications since it was discovered in 2008 [38]. Cassidy-Stone et al. has reported that over 23,100 compounds were screened on yeast growth (primary screen) followed by subsequent screening of effects on mitochondrial morphology (secondary screen) [36]. Investigators have found the inhibiting effects of Mdivi-1 on Dnm1 and mammalian homolog Drp1 [39]. Instead of noncompetitively, Mdivi-1 combining with Drp1 suppress the GTP hydrolysis just like the general inhibitor Dynasore. Besides, Mdivi-1 selectively inhibits Drp1 by binding to an allosteric site and block self-assembly and the recruitment of Drp1 to the mitochondria, attenuating mitochondrial fission [40, 39].

The inhibiting activity of Mdivi-1 to Drp1 GTPase can reverse the promotive effects of mitochondrial fission on HCC behaviors. Mutation of tumor suppression gene TP53 is universally acknowledged as a characteristic of HCC [41]. Zhan et al. reported that increased mitochondrial fission augments proliferation of HCC by facilitating the G1/S phase transition. Decreased expressions of p53 and p21 are also observed. While p65, cyclin D1, and cyclin E1 overexpress in tumorgenesis, fortunately, phenomenon and phenotypes can be reversed by Mdivi-1 treatment [42]. Moreover, Mdivi-1 can also interfere with the crosstalk between the NF-*κ*B and TP53 pathways. Activation of the NF-*κ*B signal pathway occurs in HCC, positively regulating expression of various targets which involved in tumor cell survival, stemness, and oncogenic functions [43]. Crosstalk between the two tumorigenesis-determined pathways is recently taken into account [44, 45]. Use of Mdivi-1 attenuate mitochondrial fission in HCC along with induction apoptosis by upregulated Bax and downregulated Bcl-xL-induced increase the permeability of the mitochondrial membrane and subsequent release of cytochrome c from the mitochondria into the cytosol [44]. Decreased autophagy is also detected due to downregulation of the ROS-mediated positive effects of mitochondrial fission on the AKT/IKK/NFKBIA/NF-*κ*B pathway and the negative on the AKT/MDM2/TP53 pathway [46]. To sum up, Mdivi-1 efficiently inhibits mitochondrial fission and downregulates HCC behaviors through targeting key protein Drp1.

### 4.2. BAPTA-Am

BAPTA-AM, 1,2-bis (*O*-aminophenoxy)ethane-*N*,*N*,*N0*,*N0*-tetraacetic acid tetrakis (acetoxymethyl ester) is a cell-permeable Ca^2+^ buffering agent, serving as a second messenger that regulates various physiological activities in cells. Ca^2+^ is essential for cell survival, but imbalance of cytosol calcium will result in diseases such as cancers [47]. Meanwhile, autophagy is a eukaryotic lysosomal bulk degradation system that delivers a cellular material to lysosomes for basal turnover and metabolism of cell components, but it can also enable survival and growth of tumor cells [48, 49]. Increasing evidences have shown that elevated [Ca^2+^]c stimulates autophagy when using Ca^2+^ chelator [50]. BAPTA-AM has been used to block autophagy by chelating cytosolic Ca^2+^ to downregulate AMPK-mediated autophagy, thus inhibiting the progression of cancers [51, 52]. Moreover, store-operated Ca^2+^ entry (SOCE) is a ubiquitous signal pathway playing important roles in homeostasis of Ca^2+^. Stromal interaction molecule 1/2 (STIM1/2) and CRCM1/ORAI1, located in the endoplasmic reticulum (ER) and cell membrane, respectively, are core components of SOCE [53]. The Ca^2+^ signal pathway such as Ca^2+^/CAMKK/AMPK and Ca^2+^/CaMKII/ERK are associated with tumor behaviors, including proliferation, migration, and autophagy [54, 55].

Recent studies have demonstrated the crosstalk between mitochondrial fission and the Ca^2+^ pathway and confirmed the value of BAPTA-AM in the treatment of HCC. Mitochondrial fission upregulates the level of [Ca^2+^]c via the STIM1-mediated SOCE signal pathway, forming a positive feedback loop, thus promoting HCC autophagy through the Ca2+/CAMKK/AMPK pathway [56]. Drp1-dependent fission promotes the binding of P65/RelA (a key subunit of NF-*κ*B) to STIM1 promotor, thus enhancing the expression of STIM1. The increasing expression of STIM1 results in the influx of Ca^2+^ into cytosol which upregulates Drp1 and Fis1 transcription factors NFATC2 and c-Myc and augments the mitochondrial fission. Therefore, a positive feedback loop has been formed in the process of HCC. In addition, the latest report has demonstrated that such a feedback loop can also activate the Ca^2+^/CaMKII/ERK/FAK pathway to promote HCC migration [57]. On this basis, the calcium signal pathway may be defined as a key direction for targeting mitochondrial fission and modulating HCC behaviors.

To investigate the possibility of targeting the positive feedback loop to control HCC progression, researchers use intracellular Ca^2+^ chelator BAPTA-AM to downregulate the calcium signal pathway in HCC (Figure 2). The results showed significantly decreased levels of fragmented mitochondrial and remarkably reversion of the overexpression of autophagy marker LC3-II in HCC, suggesting the inhibiting effects of BAPTA-AM on mitochondrial fission as well as autophagy [54]. Despite the limited numbers of publications, forceful evidences with regard to the positive feedback between Ca^2+^ and mitochondrial fission have provided a new idea for the research and treatment of HCC.

### 4.3. miR-125b

MicroRNAs are endogenous noncoding RNA molecule of 20-30-nucleotide (nt) length that target hundreds of mRNAs to mediate the expression of various human proteins associated with tumor cell processes, such as cell cycle regulation, invasion and apoptosis, play important roles in tumorgenesis [58, 59]. miR-125b belongs to the highly conserved miR-125 family and is constituted by miR-125b-1 and miR125b-2 in humans [60]. Much investigations have demonstrated that miR-125b suppresses proliferation and invasion and induces apoptosis in various cancer cells including breast carcinoma, HCC, renal cell carcinoma, and cholangiocarcinoma [61–64].

Mitochondrial protein 18 kDa (MTP18) is an internal mitochondrial membrane protein that contains three highly hydrophobic *α*-helical stretches [65]. The indispensable role of MTP18 in mitochondrial fission contributes to the maintenance of mitochondrial integrity and morphology, but it can also play a pivotal oncogenic role in cancers [66, 67]. Compelling evidence has demonstrated the suppressive effects of miR-125b on the expression of MTP18 and mitochondrial fission [68]. It is reported that miR-125b inhibits the proliferation and cell cycle progression of HCC [69]. The underlying mechanism has been unveiled that the overexpression of MTP18 can be downregulated, suggesting the promising value of miR-125b in the treatment of HCC [70].

## 5. Conclusions and Future Remarks

Molecular pathways in dynamics of mitochondrial fission is an advanced but burgeoning issue arousing wide attention in recent decades. Many have emphasized the vital functions of the mitochondria in providing majority of ATP with high efficiency through aerobic respiration and other physiological functions in the past, but increasing evidences show that imbalance of the two opposite processes occur in cells, especially fission, are related to diseases including cancers. Several studies, as listed above, have demonstrated that the potential mechanisms of HCC behaviors induced by mitochondrial fission. Drp1 serves as one of the key proteins modulating the division process, targeting Drp1-mediated fission to regulate HCC and integratedly describing related molecular networks will be of significance in future works. Studies on other proteins that occupy a decisive position in the recruitment of Drp1 can also avail the elaboration of the whole process of progression of HCC and also facilitate detection and diagnosis of HCC.

## Figures and Tables

**Figure 1:** Mechanism of mitochondrial fission. (a) Drp1 are recruited to the surface of the mitochondria from cytosol by Fis1, MFF, MiD49, and MiD51. (b) Drp1 assembles into higher-order structures, forming rings and spirals around mitochondria. (c) The spiral structures sever the mitochondria through GTP hydrolysis.

**Figure 2:** The mechanisms of Ca^2+^ positive feedback loop in HCC. Increasing mitochondrial fission activates the STIM1-mediated SOCE pathway and upregulates the level of Ca^2+^ influx, thus activating the CAMKK/AMPK and CaMKII/ERK/FAK pathways and promoting autophagy and migration of HCC. Influx of Ca^2+^ into cytosol upregulates Drp1 and Fis1 transcription factors NFATC2 and c-Myc, facilitating mitochondrial fission and forming a Ca^2+^ positive feedback loop. BAPTA-AM serves the function of HCC blocking the positive feedback loop by chelating cytosolic Ca^2+^.
